The article "Analysis on the Influence of Western Ecological Aesthetics on Environmental Design of China's “Beautiful Countryside”" was published in 2022. Journal: J Environ Public Health.

# Analysis on the Influence of Western Ecological Aesthetics on Environmental Design of China's “Beautiful Countryside”

**DOI:** 10.1155/2022/1271825

**Published:** 2022-08-16

**Authors:** Weiwei Li

**Affiliations:** The Fine Arts and Design Faculty, Xuchang University, Xuchang, Henan 461000, China

## Abstract

At this stage, the promotion of China's agricultural revitalization plan has provided new demands for the development of agricultural construction. In the process of urban and rural planning, more and more attention has been paid to the protection of rural traditional culture and aesthetic values, as well as the requirements of characteristic aesthetics. In recent years, as we pay more and more attention to the environmental protection ability and aesthetic ability of rural life, we also pay more attention to improving the rural environment, promoting rural rejuvenation, and paying attention to shaping the livable space quality of rural living environment to meet the needs of modern life and soul. “Beautiful countryside” is one of the modern development concepts explicitly put forward by China, which advocates the harmonious symbiosis aesthetic idea of “harmony between man and nature.” Building a beautiful countryside is the key point of rejuvenating the countryside, and the exploration of rural aesthetics is also the important significance of realizing the great rejuvenation goal of China's rural areas. Environmental design in the construction of “beautiful countryside” is a major decision and historical task for building a new countryside in China, and building landscape design suitable for the needs of rural development is the current requirement of social development. The article firstly analyzes the challenges and opportunities of China's “beautiful countryside” environmental construction; secondly, by digging into the philosophical ideas of deep ecology, ecological aesthetics, and the relationship between man and land in the West, it analyzes the application strategies and practical methods of these practical philosophies. It provides corresponding theoretical and practical enlightenment for my country's “beautiful countryside” environmental design strategy.

## 1. Introduction

With the gradual development of urbanization, the long-term and disorderly urbanization construction occupies a large amount of rural resources, and the rural environment is continuously damaged [1]. Unbalanced economic development has led to more and more polarization of space, resulting in widespread social and economic problems in rural areas and more “urban villages” were left and added in the city. On the one hand, the development of modern urbanization in China has encountered obstacles; on the other hand, the historical and cultural heritage of traditional villages has disappeared, the main role of traditional rural economic development has been ignored, traditional culture and modern life elements are mixed in the urban-rural fringe, and a large number of traditional cultural heritage has been destroyed [2]. This undoubtedly brings many challenges and difficulties to the construction of beautiful countryside in China. How to find a balance between towns and villages has become the main difficulty. The Ministry of Housing and Urban-Rural Development of the People's Republic of China has calculated the changing trend of the number of villages in my country from 2009 to 2017. According to the “2017 Urban and Rural Construction Statistical Yearbook Data” released by the Ministry of Housing and Urban-Rural Development, the number of villages in China in 2017 decreased to 2.449 million, a year-on-year decrease of 6.4%. Compared with 2.73 million in 2010, a decrease of 10%, as shown in Figure 1 [3]. This shows that with the intensification of modernization and the invasion of urbanization, China's rural areas are largely damaged. In addition, the environmental humanistic value and artistic value in the township construction have not been paid enough attention. With the lack of effective and scientific design and control of agricultural development in the past, and the natural change caused by investors, the contradiction between agriculture, and housing has become more and more obvious [4]. Enterprises and communities pay more attention to production and business activities in agricultural areas, and there are situations that damage the agricultural landscape, such as deforestation and land reclamation. In the process of the development and construction of traditional Chinese villages, because of the unreasonable “out of control” management of the government, the rural areas were divided into small areas. In addition, some farmers and builders neither do have a sense of rural cultural identity and aesthetic awareness, nor do they have understanding and confidence in the value of rural historical and cultural heritage, and the phenomenon of frequent destruction of historical sites and random “protection” has led to rural traditional culture. The lack of aesthetic ability and the lack of ideology that attaches great importance to traditional culture have led to the gradual disappearance of traditional aesthetic values and rural life forms passed down from generation to generation, as well as the gradual loss of folk skills and traditional customs [5]. Due to the lack of awareness of the ecological functions and aesthetic values of rural areas, many ancient town development projects cut off the core values and aesthetic connotations rooted in the historical context of rural areas, resulting in many excessive “commercialization” and cultural “homogenization” deformed town. This will make the construction of beautiful countryside, without the dominance of local characteristic culture, make the countryside become the same and lack of its uniqueness.

The central government's “13th Five-Year Plan” proposal clearly pointed out: “carry out the improvement of the rural living environment, strengthen the protection of traditional village dwellings and historical and cultural villages and towns, and build beautiful and livable villages.” “However, the majority of urban and rural builders continue to ask.” Where is the “beautiful country” and how to achieve “beautiful and livable.” Western scholars generally believe that the construction of rural areas should not be limited to spatial planning, visual design, and infrastructure construction, but should correspond to the transformation of production methods. Space for consumption and conservation [6]. During the new construction cycle, if the country still uses the old agricultural master plan in this period, or simply designs the agricultural environment from the perspective of farmers' production and living needs, it will not be able to overcome the current severe agricultural problems, but will make the existing social structure, ecological balance and economic and social development of the entire agricultural area [7]. Therefore, it is necessaryfor rural leaders to understand their eagerness for natural and culturalelements in rural ecology. At present, many western countries are developingalong a special path with challenges, that is, breaking through the urban-ruraldual pattern and promote integrated and coordinated development, which is to form a new industrial urban-rural relationshipthat promotes agriculture, cities lead the countryside, industry andagriculture benefit, and urban and rural areas integrate together. In this era full of challenges andopportunities, the western ecological aesthetics theory and the Chinese ruralecological construction experiment conducted on this basis have considerablereference value for the current construction of “beautiful villages” [8].

The construction of beautiful countryside is an important focus for rural revitalization. Rural revitalization has an aesthetic value. It is necessary to recognize the aesthetic value of the countryside and regard the countryside as an aesthetic existence. In the context of the rapid development of society and the consumption of “fast food” aesthetic culture, building a rural aesthetic system in China's new rural era is to solve the problems of lack of aesthetic awareness and weak aesthetic ability in the process of rural construction, and to establish a correct way of thinking, values and an effective way to revive the traditional rural culture.

## 2. Theoretical Technology

### 2.1. Theoretical Background

In the long historical development of our country, as well as in the development of different fine arts such as architecture, sculpture, art, music, and poetry, we can see people's requirements for beauty in aesthetic cognition and aesthetic activities, and vividly express the beauty and harmony of various periods and regions in the world. However, the crystallization of the sublimation of people's aesthetic outlook is not only pure aesthetics, but also the form of aesthetic existence in people's actual life. Chinese traditional literature mainly comes from the countryside. “Homesickness” describes people's pursuit of the beauty of the rural scenery and the simple life in the countryside. Traditional aesthetics was conceived and produced in the rural living space on the vast Chinese territory. With the gradual development and formation of rural and urban areas, people's requirements for environmental order and a better life have also been raised to a deeper level of rural aesthetics [9]. The countryside in the context of aesthetic science is an important part of the ecological system. The beauty of the countryside is a light of life, shining people on the track of sustainable development. In the world rural culture, mountain villages, with their unique natural ecological conditions and distinctive artistic characteristics, highlight the achievements of people's aesthetic innovation from ancient to modern times [10].

In recent years, with the gradual improvement of our environmental awareness and aesthetic ability of agricultural development, creating a good agricultural production environment, promoting agricultural rejuvenation, and meeting people's health and psychological requirements have been increasingly valued. “Beautiful countryside” is one of the modern construction ideas put forward by China [11]. Compared with the past, which only focused on the economic strength of rural areas to measure the development level of villages and towns, now more emphasis is placed on the transformation of rural ecological protection and the pursuit of “harmony between man and the environment.” The harmonious coexistence between man and nature refers to that man and nature are a community of life and a state of sustainable development of the relationship between man and nature. One harmonious coexistence aesthetic thought, developing the “two mountains” theory of socialist rural construction in the new era is an important development concept proposed by General Secretary Xi Jinping. In order to protect the rural ecological environment and achieve green development, the planning and construction of beautiful rural areas are imperative [12].

### 2.2. The Connotation of Traditional Rural Aesthetics

The so-called rural aesthetics is not a very advanced, “academic” art theory, but a value recognition based on regional culture and the understanding of beauty constructed based on this value identity. The traditional rural aesthetics has a unique aesthetic connotation. From the perspective of overall characteristics, traditional Chinese rural aesthetics often have the attributes of rural life, showing the natural features of the countryside and the beauty of farm life. When expounding the beauty of the countryside, ancient literati often described the natural scenes and social customs of the countryside through poetry, paintings, and other carriers and methods [13]. The traditional rural area also highlights the conservative and restrained aesthetic characteristics because it is far from the city center, and retains the traditional family oriented culture and rural ethics more. Therefore, traditional rural aesthetics contains a kind of beauty of farming culture, beauty of rural landscape, beauty of scholars, and beauty of rural ethics, as shown in Figure 2.

### 2.3. The Theoretical Connotation and Historical Process of Chinese Ruralism

Chinese tryism refers to a planning concept that reflects regional economic development, urbanization of infrastructure, and environmental landscape between cities and the countryside. The development process of Chinese ruralism can be roughly divided into three stages, as shown in Table 1, namely, ancient simple ruralism, modern ruralism, and modern new ruralism. (1) The simple rural theory in ancient China originated from the ancient Chinese society and agricultural civilization, which fully emphasized the establishment of rural economic infrastructure. The rural management methods also reflected the important role and significance of moral ethics and blood relationship in the social and political development of China. (2) The general characteristic of rural socialism in China since modern times is that agricultural development is regarded as a backward social field that needs reform. From various agricultural development experiences in the period of the Republic of China to the land reform in the period under the control of the Communist Party, how to carry out the rural revolution through agricultural reform. Activities to revitalize the countryside. 3) In the new era environment, with the change and development of rural positions and values, modern rural socialist ideas have produced various forms of rural construction practices and corresponding ideas [14].

## 3. Theoretical Research on the Construction of Beautiful Countryside based on Ecological Aesthetics

### 3.1. Understand the Logical Starting Point of Beautiful Rural Construction from the Time Dimension

Aesthetic thought is a kind of abstract understanding of beauty with strong subjectivity. It is the cohesion of people's ability to understand beauty and aesthetic evaluation ability, which integrates personal thoughts, feelings, and aesthetic preferences, and generally fully embodies the aesthetic ideal of The Times and the aesthetic temperament of society. Aesthetic thought is not only a simple thought or artistic ideology but also a thinking method integrating art, society, and humanity, with political, economic, and cultural characteristics and functions. The development adjustment of China's leading rural development planning objectives and the change of the focus of academic discussions hide the logical progression of rural aesthetic development [15]. Therefore, we must return to the historical node in the past development process from the current reality based on the logic of historical development, reflect back to the present from the perspective of human development, and pursue the present and the aesthetic significance of the past and the future in the nostalgia and progress of the countryside. The logical starting point of rural aesthetics is shown in Figure 3.

Since the period of agricultural revitalization in the 1920s and 1930s and the formulation of the current national agricultural revitalization policy, China's strategic agricultural development policy has been adjusted from farmland, housing, and transportation construction to environmental governance, rural scenery protection, and leisure tourism, and so on. In 2020, China will introduce an important policy of comprehensively rejuvenating Chinese traditional culture, and the construction of “beautiful villages” will also be one of the important tasks in the integration and development of Chinese culture. Therefore, the current concept of “rural beauty” is a major demand for national policy guidance in the process of new rural construction and development. As shown in Table 2, the ecological civilization concept of the “twin mountains” theory directly explains the important theory of contemporary American Rural aesthetics [16].

### 3.2. The Extension of Multidisciplinary Theory in the Construction of Beautiful Rural Environment

Through the discussion in the last part, we can realize the process of rural aesthetic theory in the construction of a beautiful countryside. However, rural aesthetic theory is not a field worth exploring, and it is a multidisciplinary complex. Rural renewal is a major global issue. It should be the main component of the theoretical research on environmental protection art, natural art, landscape art, community art, economic art, engineering art, and settlement art, as shown in Figure 4. Ecological aesthetics is an important aesthetic theoretical basis for the construction of rural ecological civilization, and the proposal of rural aesthetics is an extension of ecological aesthetics research in the dimension of rural areas. The core principles of ecological holism he proposed laid the foundation for the ecological holistic macro vision and way of thinking for the construction of ecological civilization.

In the field of ecological aesthetics, Mr. Zeng proposed “ecological ontology aesthetics.” Under the great historical background of the vigorous development of China's rural art, China's rural development should be guided by the development of China's rural art from the perspective of ecological aesthetics, explore the overall aesthetic relationship between people and rural areas, and change the current non aesthetic problems in rural areas so as to achieve the aesthetic and living state of people and rural areas in accordance with the ecological laws [17]. It is a dynamically balanced, harmonious, and healthy rural aesthetic concept that one's urban and rural development develops under the natural aesthetic conditions, and contains the ultimate concern for people's future destiny.

### 3.3. Basic Elements and Structural Analysis of Beautiful Rural Construction

A village is a complex composed of natural basic elements such as mountains, fields, and rivers, artificial environmental elements such as buildings, roads, environmental sketches, and squares, and human environmental elements such as concepts, beliefs, and cultural relics. “The consistency of human and material nature (cosmic level),” is which the objective material elements and human aesthetic subjective feelings jointly constitute the basic elements of rural beauty, and are the most important component of building a beautiful rural area [18]. In order to promote the effective implementation of the rural revitalization policy and better guide and promote the construction of beautiful villages in China, China has also issued the evaluation of beautiful rural development, as shown in Figure 5.

Under the background of the establishment of the evaluation index system of “beautiful countryside” planning and construction, the elements of contemporary rural aesthetics are extracted and summarized, and the aesthetic factors such as the sky, the landscape, the vegetation, the texture, the streets, the roads, the buildings, and the public services of the countryside are passed through a certain aesthetic method. By integrating with the effect, Table 3 shows the road construction in each region of the country in the construction of beautiful villages [19]. Based on this, establishing and refining the evaluation content and evaluation standards of contemporary rural aesthetics will help to further deepen and improve the beautiful rural evaluation system. By strengthening the rural core elements and softening the rural boundary elements, the structural optimization method protects the rural characteristics from being homogenized by the city, and the outer edge of the rural area is more open so that the rural area can achieve sustainable development in the new urban-rural integration relationship. Therefore, the exploration and integration of contemporary rural aesthetic elements can also improve the basic elements of rural areas, reduce the marginal factors, thus enhancing the cohesion of rural areas and promoting the common growth of urban and rural areas.

### 3.4. Reconstruction of the Structural Frame of Aesthetic Space in the Construction of Beautiful Rural Environment

The aesthetic structure of the countryside includes the aesthetic theme and aesthetic object in the countryside, and has a unique aesthetic structure and aesthetic realm. In reality, the theme and object of aesthetics are related to each other, and they are consistent in the perceptual world, raising the freedom and comfort beyond practicality and utility to the height of image. Therefore, the structure of rural aesthetic space is not only confined to the biological form, but also has a deeper spiritual foundation and spiritual characteristics. Therefore, the structural framework of rural aesthetic space must have a structural framework and characteristics that are connected and supported by three levels: material structure, spiritual structure and spiritual structure, as shown in Figure 6. The material structure space includes the materialized space composed of the contemporary rural aesthetic requirements and the traditional aesthetic forms; the human space structure includes the spiritual space structure composed of policy system, cultural and educational content, social values and aesthetic taste; the psychological structure is produced in the process of determining and evaluating the value of aesthetic space and artistic conception space in rural areas [20].

## 4. The Predicament of “Beautiful Countryside” Environmental Design and the Enlightenment of Western Ecological Aesthetics to Environmental Design

### 4.1. Analysis of the Predicament of “Beautiful Countryside” Environmental Design

#### 4.1.1. Emphasis on Economic Development and Light on Aesthetic Design

China's current urban construction policy objective is “applicable, economic, green and beautiful.” Although this policy fully considers the requirements of urban ecology and aesthetics, in the practical operation of urban and rural construction, it often pays more attention to application and economy, and sometimes even is applied. It is divided and even opposed to economy, green, and aesthetics. At the same time, the research on the beautiful countryside in China is mainly rooted in the fields of economic and social development, public management, and urban and rural planning, while less attention is paid to the creation of aesthetic characteristics of rural landscape. However, if rural beauty has no aesthetic value, what is the word “beautiful”

#### 4.1.2. Emphasis on the City and Less on the Countryside

In the process of China's high-speed urbanization, there are also regional differences and urban-rural differences in different degrees. The development, vitality, and attraction of many villages are not enough. Many middle-aged and young people prefer to leave their hometown and go to the city. The countryside has become a forgotten corner for the left behind children and the elderly. In addition, the state and society are more inclined to preferential policies for urban construction than focusing on the optimization of rural construction. To find effective means and methods to shorten the distance between urban and rural construction in China, we cannot bypass the natural function and artistic value of rural ecology, so that all farmers can feel the beautiful environment. The harmonious rural atmosphere makes everyone's nostalgia become “beautiful” nostalgia.

#### 4.1.3. Emphasis on Short-Term Interests over Sustainable Development

Under the above dilemmas, the report of the 18th National Congress of the Communist Party of China clearly pointed out: “Strive to build a beautiful China and realize the sustainable development of the Chinese nation.” Build a powerful modern socialist country that is prosperous, strong, democratic, culturally advanced, harmonious, and beautiful. General Secretary Xi also put forward the leading idea of “lucid waters and lush mountains are invaluable assets,” which shows the determination of the Chinese government to attach importance to sustainable development and the development of ecological civilization, and also points out the leading direction for “beautiful villages.”

### 4.2. Enlightenment of Western Ecological Aesthetics to the Environmental Design of “Beautiful Countryside” in China

#### 4.2.1. Inspiration from Deep Ecology

Deep ecology is the most important school in contemporary western radical environmentalism. Its emergence can be seen as the transformation from shallow environmental consciousness and environmental movement to deeper environmental movement. Therefore, environmental science is not simply a natural science but belongs to the field of ethics. However, because the traditional philosophy of Western Europe pays more attention to the separation between man and nature, science and technology and value, and deals with nature in a more objective and mechanized way, and even advocates that “man has the determination to conquer nature,” this also makes the industrial society of Western Europe believe that science and technology can deal with existing ecological problems. Therefore, the Western European ecological philosophy is based on the contemporary ecological ontology technology philosophy, and the deep environment is the most influential philosophical framework in this philosophical framework. Deep ecologists, mainly Norwegian thinker NAIS, attacked anthropocentrism in terms of morality, experience, reality, logic, and theory. The highest level of deep ecology is the “self-realization” of harmonious coexistence with all life, that is, human beings can realize their self-worth only when they are integrated into the relationship between the human community and the terrestrial community.

#### 4.2.2. Enlightenment of Ecological Aesthetics

Although “beauty” is an emotional cognition and lacks a unified moral and philosophical rational criterion and conclusion, from ancient times to now, “beauty” has always been respected by everyone along with “truth” and “good.“ Because people's feeling system is closely related to thinking and emotion, it shows that “beauty“ is affinity and integrity, and has the characteristics of natural integrity, diversity, and coexistence. Moreover, Foucault also reminded people that “thinking is not limited to the experience of the thinking subject or the expression of subjective thinking in the discourse, it is an action and practice.” Ecological aesthetics is a practical philosophy that explores the aesthetic relationship from the ecological perspective, and attaches importance to the ecological aesthetic relationship between man and nature, social relationship and ontology. Ecological aesthetics refers to people's aesthetic reflection on their own living conditions and the description of the aesthetic process of the ecological environment. “The beauty of existence” is a main content of ecological aesthetics. “The beauty of life” is a new type of natural ontological beauty but also a kind of beauty that is friendly to the environment and responsible to people. Its application can provide vitality for rural environmental construction. This has been confirmed in the history of rural development in European and American countries. Therefore, ecological aesthetics can also guide China to be more diversified and efficient in the construction of “socialist ecological civilization,“ and solve the environmental protection problems in the rural development of China to a certain extent.

#### 4.2.3. Enlightenment from the Relationship between Man and Land behind Ecological Aesthetics

The fundamental essence of “beauty” in “beautiful countryside“ is man and nature. Therefore, the first issue that ecological aesthetics should deal with is the relationship between man and land. It is no longer like traditional Chinese art, which puts the aesthetic theme, that is, people, in the first place. Instead, it attaches importance to the aesthetic relationship with people and society, pays aesthetic attention to the ecological environment between people and nature, and advocates the harmonious coexistence between people and nature and society. And take interest as the starting point to explore the essence of beauty. Promote the use of scientific ecological principles in environmental design and management that have a direct impact on animal and human habitats. The study of landscape ecological art in the West has highlighted the dual goals of visual beauty and ecological sustainability of habitats, and these two goals often affect each other. The best choice for conflict. The experience of western environmental art and architectural design has provided people with correct blueprints and lessons, and has a considerable impact on the design practice of China's beautiful countryside.

## 5. Conclusion

Starting from the idea of building a beautiful countryside, this paper argues that the rural ecological construction based on aesthetic theory is a new concept that conforms to the development of urban and rural culture, including rural ecology, industry, people's livelihood, and humanities. The current rural aesthetic theory system needs to be dialectically enriched and integrated on the soil of the core of Chinese traditional humanities, so as to establish a new concept paradigm that not only takes care of the planning and construction of a beautiful rural area but also can carry the most aesthetic elements of Chinese rural areas. The content involves the rural ecological landscape, the new life mode of agriculture, the traditional humanistic ethics of Chinese rural areas, and the aesthetic symbols of Chinese rural areas. Rural aesthetics is the main driving force to realize the harmonious construction of the current urban system. It is an effective way to effectively promote rural construction along a reasonable direction and form a complete and adaptive rural aesthetic concept.

Today, the function of traditional rural areas has long ceased. Western Rural builders generally believe that this should be closely related to various human factors, such as emerging social needs, environmental equity, identity recognition, cultural heritage, and community equality. Therefore, the factors to be considered by China Rural Environmental Design Institute Co., Ltd. should be multidimensional, systematic, and comprehensive. The western ecological aesthetics theory has laid a certain theoretical foundation for the environmental design of beautiful urban and rural areas in China, and has made certain expansion and corresponding supplement to the existing theories. In addition, the design planning and evaluation methods affected by this environment can also bring some enlightenment and reference to the exploration of a reasonable way of environmental protection design for “beautiful villages” in China so that the vast number of rural builders can explore the design planning and environmental protection aesthetics that meet the national conditions of China.

## Figures and Tables

**Figure 1:** The number and changes of villages in China from 2009 to 2017.

**Figure 2:** The connotation of traditional rural aesthetics.

**Figure 3:** The diachronic analysis of rural policy development and theoretical orientation.

**Figure 4:** The extension of multidisciplinary theory in the construction of a beautiful rural environment.

**Figure 5:** Analysis of evaluation elements for the construction of “beautiful countryside.”

**Figure 6:** Aesthetic space structure framework system for beautiful rural construction.

**Table 1:** The ideological forms of contemporary neo-ruralism in China.

Form	Position	Ideological	Characteristics
Nationalist new ruralism	Dominant ideology	Back to the country's stance	Transform the countryside, promote the modernization of the country
Developmental neo-ruralism	Transition from developmentalism	From advocating industrialization, urbanization, and labor transfer of the country to accepting ruralism	Modernize
Populist new ruralism	An important force to promote the new ruralism trend	Advocate for the necessity of the existence of the smallholder economy and the social and cultural value of the village	Promoting rural development and returning to the rural standpoint
Postmodern neo-ruralism	The main driving force of the rural construction movement	Criticize industrialization, urban environmental pollution, depoliticized and romantic	Actively build “beautiful countryside”

**Table 2:** Development of relevant rural policies in recent years.

Policy content	Focus	Policy source	Time
“Beautiful village”	Ecological construction, protect environment, comprehensive governance	“The Central Committee of the Communist Party of China and the State Council on Accelerating the Development of Modern Agriculture to further enhance the vitality of rural development Opinions,” “Central No. 1 Document”	Year 2013
New urbanization	Renovating the living environment	“National New Urbanization Plan (2014–2020)year)”	Year 2014
Construction of ecological civilization	Respect for nature, conform to nature, protect nature	“The Central Committee of the Communist Party of China and the State Council on Accelerating the Promotion of Ecological, Opinions on Civilization Construction”	Year 2015
Pastoral complex	Modern agriculture, leisure travel pastoral community	Highlight measures for the development of new rural industries, “Central No. 1 Document”	Year 2017
Rural revitalization	Prosperous industry, ecologically livable, rural culture, and effective governance rich life	The report of the 19th national congress of the communist party of China, the central committee of the communist party of China	Year 2017
		The central committee of the communist party of China and the state council issued the “Strategic Plan for Rural Revitalization (2018–2022)”	Year 2018
Rural living environment improvement	Building beautiful and livable villages	“Three-Year Action Plan for Rural Living Environment Improvement”	Year 2018
Integrate into production and life	Strengthen “beautiful countryside,” cultural construction	“Opinions on Implementing the Project of Inheritance and Development of Chinese Excellent Traditional Culture”	Year 2019

**Table 3:** The average proportion of road construction in the national beautiful rural construction /%.

Road type	Area	Fully hardened (asphalt/asphalt, cement)	Semihardened (gravel, gravel)	Unhardened (plain soil)
Farmland roads with a width of more than 3 m	Northeast, inner Mongolia	40.5	20.6	36.8
	North China	34.9	17.2	40.0
	East China	52.2	23.5	22.7
	Central China and south China	36.7	9.1	50.0
	Northwest, southwest	35.5	12.0	47.6

Farmland roads with a width of less than 3 m	Northeast, inner Mongolia	22.5	25.3	51.8
	North China	32.8	16.1	50.6
	East China	50.9	20.8	27.6
	Central China and south China	30.3	11.2	58.5
	Northwest, Southwest	20.5	16.3	61.6

## Data Availability

The labeled dataset used to support the findings of this study is available from the corresponding author upon request.
